The article "Cortisol as a Prognostic Marker of Short-Term Outcome in Chinese Patients with Acute Ischemic Stroke" was retracted in 2022. Reasons: duplicate publication; signs of a paper mill.

# Cortisol as a Prognostic Marker of Short-Term Outcome in Chinese Patients with Acute Ischemic Stroke

**DOI:** 10.1371/journal.pone.0072758

**Published:** 2013-09-12

**Authors:** Wen-Jie Zi, Jie Shuai

**Affiliations:** Department of Neurology, Xin Qiao Hospital, Third Military Medical University, Chongqing, P. R. China; University of Münster, Germany

## Abstract

**Background:**

Early prediction of outcome is important for allocation of therapeutic strategies. Endocrine alterations of the hypothalamus–pituitary–axis are one of the first stress-induced alterations after cerebral ischemia. We therefore evaluated the prognostic value of serum cortisol in Chinese patients with an acute ischemic stroke.

**Methods:**

In a prospective observational study, serum cortisol was measured using a solid-phase, competitive chemiluminescent enzyme immunoassay on admission in serum of 226 consecutive Chinese patients with an acute ischemic stroke. The prognostic value of serum cortisol to predict the functional outcome, mortality within 90 days, was compared with clinical variables (e.g., advanced age and the National Institutes of Health Stroke Scale [NHISS] score) and with other known predictors.

**Results:**

Patients with a poor outcome and nonsurvivors had significantly increased serum cortisol levels on admission (P<0.0001, P<0.0001). There was a positive correlation between levels of cortisol and the NIHSS (r = 0.298, P<0.0001), glucose levels (r = 0.324, P<0.0001) and infarct volume (r = 0.328, P<0.0001). Cortisol was an independent prognostic marker of functional outcome and death [odds ratio 3.44 (2.58–6.23) and 4.21 (1.89–9.24), respectively, P<0.0001 for both, adjusted for age, the NIHSS and other predictors] in patients with ischemic stroke. In receiver operating characteristic curve analysis, cortisol could improve the NIHSS score in predicting short-term functional outcome (Area under the curve [AUC] of the combined model, 0.87; 95% CI, 0.82–0.92; P = 0.01) and mortality (AUC of the combined model, 0.90; 95% CI, 0.84–0.95; P = 0.01).

**Conclusion:**

Cortisol can be seen as an independent short-term prognostic marker of functional outcome and death in Chinese patients with acute ischemic stroke even after correcting confounding factors. Combined model can add significant additional predictive information to the clinical score of the NIHSS.

## Introduction

In China, approximately 1.6 million stroke patients will die every year, which has exceeded heart disease to become the second leading cause of death and adult disability [1]. In addition, China has 2.5 million new stroke cases each year and 7.5 million stroke survivors [2]. Reliable prognostic markers available during the initial phase after acute stroke may aid clinical decision-making and allocation of healthcare resources.

The article "Cortisol as a Prognostic Marker of Short-Term Outcome in Chinese Patients with Acute Ischemic Stroke" was retracted in 2022. Reasons: duplicate publication; signs of a paper mill.

Numerous clinical variables (e.g., advanced age and symptom severity) have been identified as potential predictors of outcome. However, the need to identify better biomarkers as predictors of outcome in acute stroke still exists. The period following ischemic stroke can be considered as a reaction to a stressful event. The major characteristic of the stress response is the activation of the sympathetic nervous system (SNS) and the hypothalamo–pituitary–adrenal (HPA) axis [3]. In cerebral ischemia, endocrine changes of the HPA axis are one of the first measurable alterations [4]. Cortisol is a HPA axis-related hormone with a robust circadian rhythm where levels typically peak in the morning hours and decline across the day [5].

Cortisol has an important effect on the glucose, protein and fat metabolism and cardiovascular reactivity [6]. Some studies showed that high cortisol level was associated with decreased physical function [7], level of consciousness [8]. Fiorentino et al [5] reported that saliva levels of cortisol can be seen as a useful biological marker for identification of patients who are “at risk” of lower benefits from inpatient rehabilitation services. In addition, increased concentrations of cortisol have been observed in subarachnoid haemorrhage [9], and acute ischemic stroke [4]. Some studies have found that elevated plasma or urinary cortisol concentrations in acute ischemic stroke are related to greater stroke severity, larger infarct volume and/or unfavorable outcome, including death [4], [10]–[13]. For patients after acute ischemic stroke, high serum cortisol level was significantly correlated to the presence of acute confusional state [8]. We propose a hypothesis that higher levels of serum cortisol at admission could predict short-term outcomes in Chinese patients with acute ischemic stroke. The aim of this prospective cohort study was to verify this hypothesis.

## Subjects and Methods

### Patients and Study Design

We conducted a prospective cohort study at the neurology department of the General Hospital, Tianjin Medical University, China. From February 2009 to September 2012, all patients with first-ever acute ischemic stroke were included. All patients were Chinese. All patients were admitted within 48 hours of experiencing a new focal or global neurological event. Brain imaging (either CT or MRI) was performed routinely within 24 to 48 hours after admission. An acute ischemic stroke was defined according to the World Health Organization criteria [14]. We excluded patients with other causes of activation of the HPA axis (eg, those with surgical procedures within the last 3 weeks or those with concomitant preexisting or nosocomial infections), intracranial hemorrhage, malignancy, febrile disorders, acute or chronic inflammatory disease at study enrollment. Patients receiving immunosuppressive agents, all types of steroids, and psychotropic drugs were also excluded.

The article "Cortisol as a Prognostic Marker of Short-Term Outcome in Chinese Patients with Acute Ischemic Stroke" was retracted in 2022. Reasons: duplicate publication; signs of a paper mill.

One hundred healthy people matched for age and gender were assigned to the normal control group. Records of potential controls were reviewed by a neurologist (not an author) to exclude the presence of stroke, other types of diseases. Controls receiving immunosuppressive agents, all types of steroids, and psychotropic drugs also should be excluded. The Institutional Review Committee on Human Research of Tianjin Medical University approved the study protocol. The patients or their relatives gave written informed consent prior to entering the study.

### Clinical Variables

At baseline, demographic data (age and sex) and history of conventional vascular risk factors (hypertension, diabetes mellitus, atrial fibrillation, hyperlipidemia, smoking habit, alcohol abuse) were obtained. All these information were obtained through interviews. Routine blood and biochemical tests, ECG, and a baseline brain CT/MRI scan were performed in all patients at admission. Stroke severity was assessed on admission using the National Institutes of Health Stroke Scale (NIHSS) by a neurologist [15]. The NIHSS score ranges from 0 to 34 and higher values reflect more severe neurological damage. Whenever the NIHSS values were missing, values were estimated from chart review retrospectively, previously shown to give reliable estimates for NIHSS [16]. Stroke subtype was classified according to TOAST (Trial of Org 10172 in Acute Stroke Treatment) criteria [17]. The clinical stroke syndrome was determined by applying the criteria of the Oxfordshire Community Stroke Project: total anterior circulation syndrome (TACS); partial anterior circulation syndrome (PACS); lacunar syndrome (LACS); and posterior circulation syndrome (POCS) [18].

### End Points and follow-up

We also recorded time from symptom recognition to admission. We considered the following endpoints: (i) the primary end-point was functional outcome on day 90. Functional outcome was assessed by the modified Rankin Scale (mRS) [19]. A favourable functional outcome was defined as a mRS of 0–2 points, whereas an unfavourable outcome was defined as a mRS of 3–6 points; (ii) secondary end-points were all-cause mortality within 90 days. Outcome assessment was performed by one trained medical staff blinded to cortisol levels with a structured interview, if discharged, with telephone interview.

The article "Cortisol as a Prognostic Marker of Short-Term Outcome in Chinese Patients with Acute Ischemic Stroke" was retracted in 2022. Reasons: duplicate publication; signs of a paper mill.

### Neuroimaging

MRI with diffusion-weighted imaging (DWI) was available in 152 stroke patients (67.2%). In those patients, DWI lesion volumes were determined by one experienced neurologist unaware of the clinical and laboratory results. The infarct volume was calculated by using the formula 0.5×*a*×*b*×*c* (where *a* is the maximal longitudinal diameter, *b* is the maximal transverse diameter perpendicular to *a* and *c* is the number of 10-mm slices containing infarct) [20].

### Blood Collection and Quantification

Blood samples of patients and controls were obtained at 6:00 AM in the next morning of the day of admission. After centrifugation, aliquots of the samples were immediately stored at −80°C before assay. Serum cortisol concentration was measured with a solid-phase, competitive chemiluminescent enzyme immunoassay in a calibrated IMMULITE 2000 analyzer (Diagnostic Products Corporation, Los Angeles, CA, USA).The normal range of morning serum cortisol concentration in our hospital laboratory is 145 to 650 nmol/L, which is broadly the same as that of other laboratories (201–681 nmol/L [21], 138–690 nmol/L [22], 119–618 nmol/L [12]).The detection limit was 5 nmol/L. The intra-assay coefficient of variation [CV] and inter-assay CV were 1.5–3.2%, 2.1%–4.3%, respectively. For all measurements, levels that were not detectable were considered to have a value equal to the lower limit of detection of the assay

### Statistical Analysis

Results are expressed as percentages for categorical variables and as medians (interquartile ranges, IQRs) for the continuous variables. Proportions were compared using the χ2 test, and the Mann–Whitney test to compare continuous variables between groups. Correlations were determined using Spearman critical value rankings. Multivariate analysis was performed by binary logistic regression analysis, which allows adjustment for confounding factors (age, stroke syndrome, stroke etiology, the NIHSS score, infarct volume, vascular risk factors, glucose and C-reactive protein). Results were expressed as adjusted OR (odds ratios) with the corresponding 95% CIs (confidence intervals). Receiver operating characteristic (ROC) curves were utilized to evaluate the accuracy of cortisol to predict outcomes and death. Area under the curve (AUC) was calculated as measurements of the accuracy of the tests. The AUC summary equals the probability that the underlying classifier will score a randomly drawn positive sample higher than a randomly drawn negative sample. The time to death was analyzed by Kaplan–Meier survival curves. Two-sided P values of less than 0.05 were regarded as significant. All statistical analysis was performed with SPSS for Windows, version 20.0 (SPSS Inc., Chicago, IL, USA).

The article "Cortisol as a Prognostic Marker of Short-Term Outcome in Chinese Patients with Acute Ischemic Stroke" was retracted in 2022. Reasons: duplicate publication; signs of a paper mill.

## Results

### Baseline characteristics of study samples

During the inclusion period, 313 patients were registered. Acute ischemic stroke was diagnosed in 237 patients (45 with transient ischemic attack, 4 with haemorrhagic stroke, 10 with onset of symptoms >48 hours, 7 without informed consent, 4 with systemic infections, 3 with malignant tumor and 3 with surgical procedures within the last 3 weeks were not analyzed) and 226 completed follow-up (8 lost to follow-up and 3 withdraw). In the study population, 149 (65.9%) were male and median age was 65 years (interquartile ranges,IQR 55–74). The median time from symptom recognition to admission to hospital was 6.5 hours (IQR 2.5–11.5), and 198 patients (87.6%) were admitted within 24 hours of symptom recognition. The median NIHSS score on admission was 6 points (IQR, 3 to 10). Hypercortisolemia was found in 64 (28.3%) patients. An unfavorable functional outcome was found in 77 patients (34.1%) with a median mRS score of 4 (IQR, 3–6). 34 patients died, thus the mortality rate was 15.0%. The baseline characteristics of the 226 patients presenting with acute ischemic stroke are described in Table 1.

**Table 1:** Baseline characteristics of acute ischemic stroke patients.

Characteristics	All	Good outcomes	Poor outcomes	p^a^
	(n = 226)	(n = 149)	(n = 77)	
Male sex (%)	149(65.9)	99(66.4)	50(64.9)	NS
Age (years), median(IQR)	65(55–74)	61(50–68)	74(62–79)	<0.001
Stroke severity, median NIHSS score (IQR)	6(3–10)	3(2–7)	10(6–15)	<0.001
Infarct volume(mL,IQR; n = 152)	9(5.8–17)	8(4–12)^b^	12.5(8.3–65)	<0.001
Vascular risk factors no. (%)				
Hypertension	169(74.8)	105(70.5)	58(83.1)	<0.01
Diabetes mellitus	63(27.9)	40(26.8)	23(29.9)	NS
Hypercholesterolemia	59(26.1)	43(28.9)	16(20.8)	<0.01
Coronary heart disease	66(29.2)	44(29.5)	22(28.6)	NS
Atrial fibrillation	49(21.9)	34(22.8)	15(19.5)	NS
Family history for stroke	55(24.3)	39(26.2)	16(20.8)	NS
Smoking habit	52(23.1)	36(24.2)	16(20.8)	NS
Alcohol abuse	48(21.3)	32(21.5)	16(20.8)	NS
Clinical findings median(IQR)				
Systolic blood pressure(mmHg)	156(145–177)	155(143–174)	158(147–180)	NS
Diastolic blood pressure(mmHg)	90(82–99)	88(81–96)	91(84–100)	NS
Temperature (°C)	36.9(36.3–37.5)	37.0(36.4–37.5)	36.9(36.5–37.7)	NS
BMI (kg m^−2^)	25.6(23.4–27.2)	25.5(23.3–27.0)	25.6(23.5–27.7)	NS
Heart rate (beats min^−1^)	81(69–90)	80(69–89)	81(70–90)	NS
Laboratory findings (median, IQR)				
Cortisol (nmol L^−1^)	454(389–630)	441(367–511)	643(456–786)	<0.001
Total cholesterol (mmol L^−1^)	4.11(3.41–4.94)	4.07(3.35–4.92)	4.13(3.44–4.99)	NS
HDL (mmol L^−1^)	1.31(1.05–1.63)	1.30(1.05–1.62)	1.31(1.07–1.66)	NS
LDL (mmol L^−1^)	2.10(1.37–2.71)	2.11(1.38–2.71)	2.10(1.36–2.71)	NS
Triglycerides(mmol L^−1^)	1.42(1.05–1.88)	1.37(1.06–1.72)	1.47(1.05–2.16)	NS
Glucose(mmol L^−1^)	5.62(4.99–6.93)	5.39(4.91–6.45)	6.06(5.12–7.59)	<0.01
C-reactive protein (mg L^−1^)	4.1(3.2–8.4)	3.8(3.0–7.8)	4.4(3.5–8.9)	<0.01
Leucocyte count (×10^3^ m L^−1^)	8.4(6.2–9.7)	8.3(6.1–9.4)	8.4(6.4–9.8)	NS
Stroke syndrome no. (%)				
TACS	27(11.9)	8(5.4)	27(24.7)	<0.001
PACS	87(38.5)	59(39.6)	87(36.4)	NS
LACS	45(19.9)	28(18.8)	17(22.1)	NS
POCS	67(29.7)	50(33.6)	17(22.1)	<0.01
Stroke etiology no. (%)				
Small-vessel occlusive	42(18.6)	29(19.4)	13(16.9)	NS
Large-vessel occlusive	44(19.5)	30(20.1)	14(18.2)	NS
Cardioembolic	85(37.6)	60(40.3)	25(32.3)	NS
Other	14(6.2)	7(4.7)	7(9.1)	NS
Unknown	41(18.1)	27(18.1)	14(18.2)	NS

IQR, interquartile range; TACS, total anterior circulation syndrome; LACS, lacunar syndrome; PACS, partial anterior circulation syndrome; POCS, posterior circulation syndrome; NIHSS, National Institutes of Health Stroke Scale; BMI, Body mass index; HDL, High-density lipoproteins; LDL, Low-density lipoproteins.

a *p* value was assessed using Mann-Whitney *U* test or χ2 test.

b 104 patients were with good outcomes.

The article "Cortisol as a Prognostic Marker of Short-Term Outcome in Chinese Patients with Acute Ischemic Stroke" was retracted in 2022. Reasons: duplicate publication; signs of a paper mill.

### Serum cortisol levels and stroke characteristics

The results indicated that the serum cortisol levels were significantly (p<0.0001) higher in acutely ischemic stroke patients as compared to normal controls (456; IQR, 397–621 nmol/L and 424; IQR, 368–515 pmol/L, respectively; Figure 1.). Cortisol levels increased with increasing severity of stroke as defined by the NIHSS score. There was a positive correlation between levels of cortisol and the NIHSS (r = 0.298, P<0.0001; Figure 2a.) and glucose levels (r = 0.324, P<0.0001; Figure 2b.) There was a modest correlation between levels of serum cortisol levels and age(r = 0.157, P = 0.021). There was no correlation between levels of serum cortisol levels and sex (P = 0.230). C-reactive protein and white blood cells count were not correlated with the serum cortisol levels (p = 0.103 and p = 0.124, respectively). In patients for whom MRI data were available (n = 152), there was a positive correlation between levels of cortisol and the infarct volume (r = 0.328, P<0.0001; Figure 2c.) In addition, cortisol values were significantly higher in patients with TACS 625 nmol/L (IQR 478–812) compared with patients with PACS 487 nmol/L (IQR 356–614, P<0.001), LACS 438 nmol/L (IQR 344–613, P<0.001) or POCS 476 nmol L (IQR 335–661, P<0.001). Cortisol levels were not correlated with the C-reactive protein and Leucocyte count.

**Figure 1:** Serum cortisol levels in acute ischemic stroke patients and control group. Mann–Whitney U-test. All data are medians and in-terquartile ranges (IQR). Significantly higher in stroke patients as compared to normal cases (P<0.0001).

The article "Cortisol as a Prognostic Marker of Short-Term Outcome in Chinese Patients with Acute Ischemic Stroke" was retracted in 2022. Reasons: duplicate publication; signs of a paper mill.

**Figure 2:** Correlation between serum cortisol levels and others predictors. (a) Correlation between the National Institutes of Health Stroke Scale (NIHSS) and serum cortisol levels. (b) Correlation between the serum glucose and cortisol levels. (c) Correlation between the infract volume and serum cortisol levels.

### Serum cortisol levels and outcome

Serum cortisol levels in patients with a poor outcome were significantly greater than those in patients with a good outcome (643 [IQR, 456–786] vs 441 [IQR, 367–511] nmol/L; p<0.0001; Figure 3.). In univariate logistic regression analysis, we calculated the ORs of log-transformed cortisol levels as compared with the NIHSS score and other risk factors as presented in Table 2. With an unadjusted OR of 5.98 (95% CI, 3.63–10.52), cortisol had a strong association with functional outcome. After adjusting for all other significant outcome predictors, cortisol remained can be seen as an independent outcome predictor with an adjusted OR of 3.44 (95% CI, 2.58–6.23). In addition, age, glucose level, infarct volume, and the NIHSS score remained significant outcome predictors (Table 2).

**Figure 3:** Serum cortisol levels in acute ischemic stroke patients with good and poor outcomes. Mann–Whitney U-test. All data are interquar-tile ranges (IQR). Significantly higher in poor as compared to good group (P<0.0001).

**Table 2:** Univariate and multivariate Analysis.

Parameter	Univariate Analysis			Multivariate Analysis		
	OR^a^	95% CI^a^	*P*	OR^a^	95% CI^a^	*P*
Predictor: functional outcome						
Cortisol (increase per log unit)^b^	5.98	3.63–10.52	<0.0001	3.44	2.58–6.23	<0.0001
Age (increase per unit)	1.36	0.85–2.18	0.031	1.54	0.83–2.89	0.012
NIHSS (increase per unit)	1.23	1.06–1.45	<0.0001	1.30	1.14–1.47	<0.0001
Glucose (increase per unit)	1.19	1.04–1.36	0.012	1.10	0.92–1.31	0.030
CRP (increase per unit)	1.23	1.06–1.45	0.008	1.16	1.11–1.23	0.021
Infarct volume(increase per unit)	1.11	1.00–1.22	0.006	1.13	0.87–1.31	0.002
Predictor: death						
Cortisol (increase per log unit)^b^	10.32	5.68–18.45	<0.0001	4.21	1.89–9.24	<0.0001
Age (increase per unit)	1.42	0.99–1.87	0.023	1.34	1.08–1.99	0.043
NIHSS (increase per unit)	1.52	1.14–2.99	<0.0001	1.42	0.95–2.07	0.027
Glucose (increase per unit)	1.33	1.12–1.68	0.003	1.33	0.88–2.07	<0.0001
CRP (increase per unit)	1.29	1.08–1.65	0.011	1.12	0.98–1.56	0.016
Infarct volume(increase per unit)	1.19	1.02–1.54	0.007	1.06	1.04–1.09	<0.0001

a Note that the odds ratio corresponds to a unit increase in the explanatory variable.

b This corresponds to an increase per unit of the log transformation of cortisol (thus, a log-transformed increase of 1 corresponds to a cortisol increase of 10 nmol/L).

The article "Cortisol as a Prognostic Marker of Short-Term Outcome in Chinese Patients with Acute Ischemic Stroke" was retracted in 2022. Reasons: duplicate publication; signs of a paper mill.

OR, odds ratio; CI, confidence interval; CRP, C-reactive protein; NIHSS, National Institutes of Health Stroke Scale.

The area under the receiver operating characteristics (ROC) curve to predict outcome for cortisol with an AUC of 0.78 (0.71–0.85) was in the range of the NIHSS with an AUC of 0.81 (0.75–0.89) (see table 3). Cortisol had a higher prognostic accuracy as compared to glucose (AUC 0.55 (0.43–0.67), *P*<0.01), white blood count (WBC) (AUC 0.47 (0.39–0.58), *P*<0.001) and infarct volume AUC 0.69 (0.62–0.77), *P* = 0.01). Interesting, we found that combination of cortisol and NIHSS scores could improve the NIHSS scores (AUC of the combined model, 0.87; 95% CI, 0.82–0.92; *p* = 0.01). This improvement was stable in an internal 5-fold cross validation that resulted in an average AUC (standard error) of 0.81 (0.036) for the NIHSS and 0.87(0.028) for the combined model, corresponding to a difference of 0.06 (0.014).

**Table 3:** Receiver operating characteristics curve analysis.

Parameter	Functional outcome at 90 days			Mortality at 90 days		
	AUC	95% confidence interval	*P*	AUC	95% confidence interval	*P*
Cortisol	0.78	0.71–0.85		0.81	0.73–0.79	
NIHSS	0.81	0.75–0.89	0.32	0.85	0.78–0.91	0.16
Infarct volume	0.69	0.62–0.77	0.01	0.76	0.67–0.84	0.04
Age	0.61	0.53–0.69	<0.01	0.54	0.43–0.66	<0.01
Glucose	0.55	0.43–0.67	<0.01	0.64	0.51–0.72	0.02
CRP	0.54	0.44–0.68	<0.01	0.57	0.49–0.67	<0.01
WBC	0.47	0.39–0.58	<0.001	0.55	0.43–0.67	<0.01
Combined score⋇	0.87	0.82–0.92	0.01	0.90	0.84–0.95	0.01

AUC, area under the curve; CRP, C-reactive protein; NIHSS, National Institutes of Health Stroke Scale; WBC, white blood cells.

⋇ including NIHSS and Cortisol.

Cortisol levels in 34 patients who died were significantly greater as compared with patients who survived (682 [IQR, 511–878] vs 438 [IQR, 384–563] nmol/L; p<0.0001). After adjustment for other parameters, cortisol level remained an independent predictor for mortality with an OR of 4.21 (95% CI, 1.89–9.24; see Table 2). Receiver operating characteristic curves indicated the greatest discriminatory accuracies for cortisol level (AUC, 0.81; 95% CI, 0.73–0.89) and the NIHSS score (AUC, 0.85; 95% CI, 0.78–0.91). Combination of cortisol and NIHSS scores also could improve the NIHSS scores (AUC of the combined model, 0.90; 95% CI, 0.84–0.95; *p* = 0.01). Again, this improvement was stable in an internal 5-fold cross validation that resulted in an average AUC (standard error) of 0.85 (0.023) for the NIHSS and 0.90(0.027) for the combined model, corresponding to a difference of 0.05 (0.018).

The article "Cortisol as a Prognostic Marker of Short-Term Outcome in Chinese Patients with Acute Ischemic Stroke" was retracted in 2022. Reasons: duplicate publication; signs of a paper mill.

The time to death was analyzed by Kaplan–Meier survival curves based on cortisol quartiles. Patients in the lowest two quartile (cortisol <397 nmol/L and cortisol between 397 and 456 nmol/L) had a minimal risk for death, in contrast with patients with levels in the highest two quartiles (cortisol between 456 and 621 nmol/L and cortisol >621 nmol/L, respectively) (p<0.0001) (See the Figure 4.).

**Figure 4:** Kaplan–Meier survival curves based on cortisol quartiles. Time to death was analysed by Kaplan–Meier curves based on cortisol quartiles.

## Discussion

Acute ischemic stroke acts as a stressor and thus stimulates the HPA axis resulting in increased glucocorticoid levels [4]. In this study, we firstly assessed serum cortisol levels with regard to their accuracy to predict functional outcome and mortality in patients with acute ischemic stroke within 90 days in Chinese population. Our main finding is that cortisol can be seen as an independent short-term prognostic marker of functional outcome and death in Chinese patients with acute ischemic stroke even after correcting for possible confounding factors. Combined model (cortisol and NHISS score) can add significant additional predictive information to the clinical score of the NIHSS. We also found that that cortisol levels increased with infarct volume, neurological deficit (assessed by the NIHSS) and the clinical stroke syndrome.

These results are in accordance with the results from other studies showing that hypercortisolemia was associated with older age, greater severity of neurological deficit, larger ischemic lesions on CT, worse prognoses (a greater disability and mortality) in stroke patients [8], [12], [23].

Age may influence serum cortisol [24]–[25]. We also found a modest positive correlation between levels of serum cortisol levels and age(r = 0.157, P = 0.021). Previous studies reported that fasting glucose level and insulin resistance increased with higher cortisol level [6]–[7].We also found that there was a positive correlation between levels of cortisol and glucose levels (r = 0.324, P<0.0001; Figure 3.). As expected, high levels of cortisol were associated with diabetes mellitus. The association may be confounded by obesity. It has been reported that cortisol correlated positively to inflammatory response after stroke, and it was suggested that cytokines modulate the cortisol response after acute stroke [11] by stimulating the HPA axis leading to increased levels of cortisol in the periphery [26]. Our findings were inconsistent with previous findings, and we did not find correlation between inflammatory response and serum cortisol levels.

The article "Cortisol as a Prognostic Marker of Short-Term Outcome in Chinese Patients with Acute Ischemic Stroke" was retracted in 2022. Reasons: duplicate publication; signs of a paper mill.

In our study, we found hypercortisolemia in 28.3% of patients with acute stroke. The frequency of hypercortisolemia in stroke patients has been reported in the range of 24%–38% [8], [12], [27]. This is very interesting because despite using different methods of assessment and the study population are not the same, a similar prevalence of hypercortisolemia was obtained, indicating a similar increase in adrenocortical output in stroke.

Whether the high serum cortisol is just an epiphenomenon to stroke severity or independently contributes to prognosis remains uncertain. A severe stroke *per se* implicates a poor outcome. However, there are several other reasons explaining unfavorable outcome in patients with higher cortisol levels. It cannot be excluded that these HPA axis-related hormones, once released, secondarily reinforce damage of hypoxic brain tissue and thereby contribute to the poor outcomes. Firstly, increased exposure to cortisol contributes to increased fat accumulation in visceral depots [28]. Hypercortisolism itself may potentiate ischemic neuronal injury, especially in hippocampal neurons [29]–[30], and the corticosterone-synthesis inhibitor, metyrapone, was able to prevent ischemia-induced loss of synaptic function in the hippocampus of rats [31]. The hippocampus has an important role in the feedback regulation of the HPA axis. Dysfunction of hippocampal might result in false HPA axis feedback, which increase cortisol and causes a vicious circle [32]. Secondly, patients with stroke and high cortisol levels are more prone to suffer from adverse cardiac events, which may lead to higher mortality rates [32]–[33]. Finally, a bad prognosis after stroke is the development of infectious disease which is related to an immune dysregulation resulting from neuroendocrine disturbance after stroke [34]. High cortisol levels are more susceptible to infections [7]. The specific mechanism needs to be further studied in population-based larger cohort studies.

Some limitations of this observational study merit consideration. First, without serial measurement of the circulating cortisol levels, this study yielded no data regarding when and how long cortisol is elevated in these patients. Second, the effects of circulating cortisol on long-term clinical outcome were not included in the study protocol, so these relationships were not examined beyond the 90-day clinical outcome. Third, we assessed all-cause mortality because classification of death in clinical practice can sometimes be difficult and unreliable [35]. Forth, this was only a preliminary study; these results need to be replicated in more prospective studies to determine whether or not they are stable and valid. If our findings are confirmed, clinicians assessing patients with acute stroke should consider measuring serum levels of cortisol routinely on admission.

The article "Cortisol as a Prognostic Marker of Short-Term Outcome in Chinese Patients with Acute Ischemic Stroke" was retracted in 2022. Reasons: duplicate publication; signs of a paper mill.

## Conclusions

Despite its inherent limitations, our study suggested that cortisol levels may reliably predict short-term prognosis at its onset in Chinese patient with acute ischemic stroke. Combined model (cortisol and NHISS score) can add significant additional predictive information to the clinical score of the NIHSS. We recommend that further studies should be carried out with respect to the mechanism between increased cortisol levels and poor outcome. If it is possible to elucidate this, the prognosis of these stroke patients might be improved.
